# The Relationship between Information Dissemination Channels, Health Belief, and COVID-19 Vaccination Intention: Evidence from China

**DOI:** 10.1155/2023/6915125

**Published:** 2023-01-30

**Authors:** Chuanwu Huang, Dongqi Yan, Shuang Liang

**Affiliations:** ^1^The School of Digital Media and Design Arts, Beijing University of Post and Telecommunication, Beijing 100088, China; ^2^The Key Laboratory of Trustworthy Distributed Computing and Service, Beijing University of Posts and Telecommunications, Ministry of Education, Beijing 100088, China; ^3^Beijing Key Laboratory of Network System and Network Culture, Beijing 100876, China

## Abstract

In the context of the ongoing global epidemic of COVID-19 and frequent virus mutations, the implementation of vaccine is the key to the prevention and control of the epidemic at this stage. In order to provide recommendations and evidence to support global epidemic prevention and control and vaccination efforts from the perspectives of health communication and individual psychological perceptions and to improve the vaccination rate of COVID-19 vaccine among appropriate populations, this study conducted a questionnaire survey in eight districts of Beijing and collected a total of 525 valid data points. A health belief model was used to examine the predictors of COVID-19 vaccination behavior, and the relationship between different COVID-19 vaccine information dissemination channels, residents' health beliefs, and propensity to vaccinate was analyzed. This study found the following: (1) among new media, interpersonal communication and traditional media communication channels, the new media channel had the largest number of audiences; (2) the personal health beliefs of audiences in the three information channels differed significantly, with the highest perceived benefits and lowest perceived barriers in the interpersonal communication channel and the highest perceived barriers in the new media communication channel; (3) the health belief model was a significant predictor, with perceived benefits and barriers being the most effective attitudinal variables for predicting vaccination intention. This study is valuable for advancing and improving vaccine communication diffusion research and promoting wider application of the health belief model and communication media in health communication topics.

## 1. Introduction

The COVID-19 global pandemic presents a new and unprecedented set of challenges, including the infodemic and information overload. According to Dr. Sylvie Briand, the WHO's Director of Global Infectious Disease Preparedness, the outbreak of COVID-19 was accompanied by an information epidemic (infodemic). When there is a flood of information, public cannot access reliable sources of information and correct knowledge [1]. In particular, the flood of information about vaccines leads people to adopt wrong health behaviors, even though vaccination is one of the most cost-effective and efficient public health interventions to prevent infectious diseases [2–4]. Combating COVID-19, therefore, requires the concerted efforts of multiple stakeholders to disseminate timely, accurate, and authoritative information through different media channels [5, 6].

There is a rich body of research on vaccination, with perspectives focused on exploring the factors and mechanisms influencing vaccination intentions and behaviors, demonstrating the vital influence of psychological attitudes on health behaviors [7–9]. However, these models are often rooted in the individual perspective and divorce individual vaccine decisions from the macrolevel social context in which they are interwoven, such as the information environment and social culture. Vaccination is part of the “broader social world” [10]. In particular, in the age of the media, ubiquitous media exposure significantly influences the public's willingness to vaccinate. Individual vaccine decisions are a complex interaction between individuals and many social factors, which are richly intertwined with the media information ecology and the sociocultural environment. Accordingly, this study incorporates media exposure as an information environment factor into vaccination analysis to explore how media exposure affects individual cognition and further influences the willingness to receive COVID-19 vaccination.

At the individual cognitive level, behavior change models widely used in health communication research include the health belief model, the social cognition model, and the theory of reasoned action [11]. The health belief model (HBM) was introduced in the 1850s by American social psychologists working in the Public Health Service and was originally used to explain people's attitudes and behaviors toward TB screening, including perceived susceptibility, perceived severity, perceived benefits, perceived barriers, engagement behaviors, and action cues [12]. The effectiveness of health belief models in predicting vaccination behavior has been widely demonstrated [13]. In the framework of the health belief model, perceived susceptibility, perceived severity, perceived benefits, and perceived barriers have shown significant relationships with health behavioral intentions [14]. Perceived susceptibility refers to an individual's perceived likelihood that an unhealthy behavior or virus will lead to health problems; perceived severity refers to an individual's perception of the severity of the physical, psychological, and social consequences of the disease and perceived severity of the adverse consequences of the disease. Perceived benefits refer to individuals' judgments about the likelihood of benefits from health behaviors, and perceived barriers refer to individuals' judgments about the likelihood of difficulties or costs in the process of implementing health behaviors, from decision-making to adoption [15]. Many studies have used the health belief model to analyze individuals' perceptions and attitudes toward viruses and vaccines, and the model is a valid theoretical model for predicting and explaining individual health behaviors [16]. Wong et al. [17] used the HBM framework to assess predictors of intention to receive the COVID-19 vaccine and found that the key constructs of the model, high perceived benefits, low perceived barriers, and high perceived susceptibility, were significantly associated with intention to receive the vaccine. Therefore, this study used HBM to analyze the dynamic process by which health information related to the Newcastle pneumonia vaccine influences vaccination intention. Based on the health belief theory, this study further explores the influence of information acceptance on behavioral decision-making during the decision-making process of COVID-19 vaccination intention. Based on the health belief model, this study further explores the influence of information reception on behavioral decision-making in the vaccination decision process for pneumoconiosis vaccination and proposes the “information channel-cognitive attitude-behavioral intention” framework. Two research questions were posed: how different health information channels affect the four dimensions of health beliefs, and whether different dimensions of health beliefs have an impact on COVID-19 vaccination intention.

Beijing was one of the first cities to experience an outbreak, and the region had a long-standing policy of mass vaccination with the COVID-19 vaccine. As of July 24, 2021, Beijing has an exemplary vaccination rate of 98.13% of the resident population aged 18 years and older [18]. Based on this, the purpose of this study is to collect questionnaire data from the vaccination population in Beijing, China, and to study the differences in audience health psychological attitudes under the influence of different COVID-19 vaccine information channels (traditional media, new media, and interpersonal communication) as well as the impact of psychological attitude differences on audience groups' vaccination intentions, in order to fill the aforementioned research gaps.

The rest of this study is organized as follows: Section 2 describes the study design, sample, and measurement methods.  Section 3 presents the descriptive statistics, reliability and validity analysis, nonparametric tests, and data analysis results of the regression analysis.  Section 4 provides a discussion, and Section 5 gives future prospects and the implementation of strategies of the study.

## 2. Materials and Methods

### 2.1. Survey Design

We conducted a 43-day anonymous questionnaire survey from March 1, 2021, to April 12, 2021. The survey was launched on the online survey-based platform Questionnaire Star (Changsha Ranxing Information Technology Co., Ltd., Changsha, China), which consists of more than 2.6 million Chinese members with factual personal information and diverse socioeconomic backgrounds, and it allows automatic logical proofreading to reduce input errors and avoid missing values. The survey area of this study covers Beijing city, suburban, and distant suburban areas. A total of eight districts, including Dongcheng District, Xicheng District, Haidian District, Fengtai District, Daxing District, Huairou District, Pinggu District, and Miyun District, were included, and a stratified sampling method was used to collect data. We asked each person to complete an online questionnaire lasting approximately 5 minutes and limited the study sample to respondents aged 18–59 years. Data from people who were not suitable for vaccination were eventually excluded. Questionnaires with missing values, invalid questionnaires, and blank questionnaires were excluded. A total of 525 valid samples were obtained, with an effective rate of 83.96%.

In this study, a questionnaire was designed based on literature analysis and model assumptions and consisted of five main parts: an introductory phrase, sociodemographic characteristics (e.g., gender, age, education level, and job nature; see Table 1 for details), main information acquisition channels, health beliefs (about the COVID-19 virus and vaccine), and COVID-19 vaccination intention.

### 2.2. Conceptual Framework

In terms of health information channels and health beliefs, Willis found that exchanging health information through a new media community can increase the perceived benefits and decrease the perceived barriers to using prescription drugs for people with arthritis [19]. Jones focused on the effect of new media channels on health beliefs and illustrated that when accessing information about their children's vaccinations, parents who used the new media as their primary information access channel tended to have lower perceived susceptibility to the virus, lower perceived benefits of vaccination, and higher perceived barriers related to vaccine side effects [20]. In contrast, Mcree et al. showed that parents who obtained information about vaccines on the new media generated more positive attitudes and beliefs about vaccination than parents who used other sources of information, and these parents perceived their children to be more susceptible to the virus in question and had lower perceived barriers to vaccines [21]. Vaccination rates are positively associated with multiple sources of information about vaccination, including healthcare providers, family members [22], newspapers, brochures, schools, and friends [23]. Vaccine intention may be fueled by health information obtained from a variety of sources, including new media such as the new media and social media platforms; there is growing concern about the role of cross-social media, for example, in public health promotion [24–27]. However, there is also great potential for harmful misinformation to spread through the new media, thus exacerbating vaccine hesitation. Therefore, this study included new media communication channels. The following research questions are therefore posed:

  Q1: How do different health information channels affect the four dimensions of health beliefs?
  H1: Individuals' perceived susceptibility to COVID-19 differs significantly among the three major information channels
  H2: Individuals' perceived severity of COVID-19 differs significantly among the three major information channels
  H3: Individuals' perceived benefits of the COVID-19 vaccine differ significantly among the three major information channels
  H4: Individuals' perceived barriers to the COVID-19 vaccine differ significantly among the three major information channels

In recent years, empirical studies based on health belief theory have focused on the medicine field [28]. Health belief models focus on individual-level perceptions and attitudes towards viruses and vaccines, influence individual health decisions, can be used as a basis for predicting health behaviors [29], and have been specified for research on a variety of noncommunicable or communicable diseases to explain vaccination intentions such as dengue, HPV, seasonal influenza, and influenza A [14, 30–33]. Gerend et al. examined the intention of U.S. women to receive the human papillomavirus (HPV) vaccine, which was approved for marketing in 2007, and identified correlates that influence HPV vaccination intention factors including health beliefs, physician encouragement to vaccinate, and the science of vaccine-related information. In terms of health beliefs, research has shown that perceived susceptibility, perceived severity, and perceived benefit are positively associated with behavioral intentions to vaccinate [34]. Friedman and Shepeard found that various perceived barriers (including concerns about vaccine safety the high cost of vaccination) were negatively associated with the intention to vaccinate [35]. Hsing et al. verified the validity of the dimensions of health beliefs as predictors of preventive action for pneumoconiosis [36].

Based on the above literature review and in the context of current COVID-19 risk, there are strong reasons to suggest that perceived benefit, perceived susceptibility, perceived barriers, and perceived severity are significant predictors of vaccination intention, and therefore, the following hypotheses are proposed:

  Q2: Whether different dimensions of health beliefs have an impact on intention to COVID-19 vaccine intention?
  H5: Perceived susceptibility (for coronavirus) positively affects COVID-19 vaccination intention
  H6: Perceived severity (for coronavirus) positively affects COVID-19 vaccination intention
  H7: Perceived benefit (for COVID-19 vaccine) positively affects COVID-19 vaccination intention
  H8: Perceived barriers (for COVID-19 vaccine) negatively affect COVID-19 vaccination intention

The final research model is shown in Figure 1.

### 2.3. Measures

#### 2.3.1. Information Dissemination Channels

New media, interpersonal communication, and traditional media communication are leading information dissemination channels. Respondents' responses were selected from “1 = interpersonal communication,” “2 = new media,” and “3 = traditional media” as the primary channels for obtaining information on the COVID-19 vaccine and further selected as a breakdown of the options. “Traditional media” included TV, radio, magazines, and newspapers; “interpersonal” included health workers, family members, friends, and the school; “new media” included websites, social media, short video platforms, and news apps.

#### 2.3.2. Health Beliefs

The health beliefs variable was measured by 16 questions with responses ranging from “strongly disagree” to “strongly agree” (1 = strongly disagree, 7 = strongly agree), mainly referring to the Patty Scale [37]. Positive aspects include (1) perceived susceptibility: the belief in susceptibility to the disease, (2) perceived severity: the belief that the disease has a negative impact on quality of life, and (3) perceived benefit: the belief that adopting the behavior will help reduce susceptibility or severity. The negative aspects are perceived barriers: the belief that there are some limitations or obstacles in adopting the behavior (see Table 2 for the specific scale).

#### 2.3.3. COVID-19 Vaccination Propensity

Acceptance of COVID-19 vaccination was measured by three items, with responses ranging from “strongly disagree” to “strongly agree” (1 = strongly disagree, 7 = strongly agree). The vaccination intention variable was mainly based on Young's scale [38] (see Table 3 for details).

### 2.4. Data Analysis

For the analysis of the data, Excel 2018 was used to create a database and clean the data, and SPSS 24 was used to process and analyze the data, using descriptive statistics, correlation analysis, regression analysis, and the Kruskal–Wallis H nonparametric test to investigate the relationship between the study population's access to information, health beliefs, and COVID-19 vaccination intention.

## 3. Results and Discussion

### 3.1. Reliability and Validity

The standardized Cronbach coefficients were used to test the reliability of “COVID-19 vaccination intention” and the four dimensions of “perceived susceptibility,” “perceived severity,” “perceived benefit,” and “perceived barriers” in the health belief model. The results of the SPSS output are shown in the following table: the Cronbach coefficients based on standardized terms for the variable “COVID-19 vaccination acceptance” and the coefficients of “perceived benefits” and “perceived barriers” were tested. In general, a coefficient greater than 0.8 indicates excellent internal consistency, between 0.6 and 0.8 indicates good internal consistency, and below 0.6 indicates poor internal consistency. The results of Cronbach's coefficient test for all four dimensions of this study's scale were >0.6, indicating that the reliability of the scale is good.

The validity analysis of “COVID-19 vaccination acceptance” was performed by exploratory factor analysis. The KMO test focuses on the correlation between the indicators to determine whether a principal component or factor analysis can be conducted. A KMO test result greater than 0.8 indicates excellent internal correlation, between 0.5 and 0.8 indicates good internal correlation, and below 0.5 indicates poor internal correlation. The results of the analysis showed that the KMO coefficients of the 3 questions on “COVID-19 vaccination acceptance” and the 16 questions on “health beliefs” were >0.6 with a significance level of *p* < 0.05 so that exploratory factor analysis could be conducted.

An exploratory factor analysis was conducted on “health beliefs” using the rotated component method, which is a credential for good or bad aggregation. The method was used to rotate four factors, and the four factors explained a total of 69.26% of the variance, with high overall validity. According to the factor loadings of the rotated items, the four factors conformed to the structure of the original scale, and factors 1, 2, 3, and 4 were named “perceived severity” (Cronbach's *α* = 0.669), “perceived susceptibility” (Cronbach's *α* = 0.885), “perceived benefit” (Cronbach's *α* = 0.874), and “perceived barriers” (Cronbach's *α* = 0.873), respectively (Table 2).

The results of the exploratory factor analysis for “COVID-19 vaccination intention” showed that the three factors of the “COVID-19 vaccination intention” dimension explained a total of 91.969% of the variance. Therefore, it was concluded that the three questions could detect “COVID-19 vaccination intention” well and had high validity (Table 3).

According to the above tests, the scale used in this study has good reliability and validity.

### 3.2. Descriptive Statistics

The results of the descriptive statistical analysis of the 525 valid questionnaires collected in this study are shown in table. The survey population covers different age groups of young, middle-aged, and old people who are suitable for vaccination; the working nature of the survey population covers “teachers and students in China,” “people who are going to work or study in medium- and high-risk countries or regions,” and “people engaged in importing cold chain, port quarantine, ship piloting, airline aircrew, fresh food, etc.” The survey population covers types of workers with high social mobility and high risk of infection and “general workers,” which meet the experimental requirements.

The new media channel is the most widely used information dissemination channel, accounting for 45.5% of the audience, while traditional media channels and interpersonal communication channels account for 29.9% and 24.2%, respectively. The audience of interpersonal communication channels as the main information dissemination channel is relatively small (Table 4).

### 3.3. Kruskal–Wallis H Nonparametric Test

The four dimensions of health beliefs are nonnormal data, so the Kruskal–Wallis H nonparametric test for independent samples is used, and the Kruskal–Wallis test for multiple independent samples can be used to analyze the significance of data differences between groups, with *p* values less than 0.05 being considered significant [39, 40].

The Kruskal–Wallis rank sum test is considered one of the most common alternative hypothesis tests, that is, if there is a difference in the treatment effect of each method, the difference is mainly reflected in the separation of the individual treatment effect measures of each group, that is, if there is a significant difference in the actual effect of these methods, then there is a ranking between the individuals tested by each method, where the rank of individuals in some methods tends to take smaller values, and the rank of individuals in other methods tends to take larger values. The following test statistic is constructed for such alternative hypotheses:

(1) $$\begin{array}{c} R_{i.}=\frac{R_{i1}+R_{i2}+...+R_{in_{i}}}{n_{i}},i=1,2,\ldots ,m\text{,}\\ R_{.}=\frac{1}{n}\overset{m}{\underset{i=1}{\sum }}\overset{n_{i}}{\underset{j=1}{\sum }}R_{ij}=\frac{n+1}{2}\text{.} \end{array}$$

*R *_*i.*_ is the mean of the rank of the “*i*” group of individuals (*i* = 1, 2,…, *m*), *R* is the overall mean. If there is a significant difference between the actual effects of these methods according to the above alternative hypothesis, then *R*_*i*_. (*i* = 1, 2,…, *m*) are more different from each other. Conversely, if H0 is true, the differences between *R*_*i*_ (*i* = 1, 2,…, *m*) should be small since the grouping is randomized. The corresponding *p* values were calculated, and when the *p* value was less than 0.05, H0 was rejected and the difference was considered large.

In this study, the data were divided into three groups based on the criteria of information reception channels, and the Kruskal–Wallis model test was applied to three groups of data from different items using SPSS to analyze whether there are differences in the four dimensions of audience health beliefs across the main information dissemination channels (Table 5).

The results of the rank mean analysis of “perceived benefits” and “perceived barriers” are shown in the table. The rank mean of “perceived benefits” under the “interpersonal communication” channel was 308.94, and the rank mean of “perceived barriers” under the “interpersonal communication” channel was 202.76. The largest proportion of the interpersonal communication options was with medical workers (including community clinics and hospitals), which accounted for 65.29%. However, the total number of cases choosing interpersonal communication as the main channel was relatively small, accounting for 24.2% of the overall sample. According to the statistical results, the rank mean of “perceived barriers” was 302.08 for the “new media” channel, which was significantly higher than that of the “interpersonal communication” and “traditional media” channel. The rank mean of “perceived barriers” is 302.08, which is significantly higher than “interpersonal communication” and “traditional media communication.” Therefore, audiences who use new media as the main information channel are more concerned about the barriers to COVID-19 vaccination, and the highest perceived barrier is “I am afraid of the side effects of COVID-19 vaccination,” which accounts for 44% of the respondents. It is necessary to further analyze whether perceived benefits and perceived barriers are significant influencing factors for the propensity to receive the COVID-19 vaccine. If both dimensions are significant influencing factors, attention should be paid to the fragmentation characteristics of online information, the possible increase of perceived barriers caused by rumors and inaccurate information, and the advantages and characteristics of interpersonal communication (Table 6).

The results of the statistical analysis answer the research questions of this study.

  Q1: How different health information dissemination channels affect the four dimensions of health beliefs?

According to the results, it can be seen that there are no significant differences in individuals' perceived susceptibility or perceived severity, but significant differences in individuals' perceived benefits and perceived barriers under the three main channels of information acquisition about the COVID-19 vaccine, namely, interpersonal communication, new media, and traditional media communication. Whether the four dimensions of health beliefs serve as key influencing factors of individual COVID-19 vaccination acceptance deserves our attention.

### 3.4. Correlation Analysis

Correlation analysis focuses on the extent to which the variables are closely related to each other, which is measured in this study using the Pearson correlation coefficient. The next correlation analysis was conducted for each research hypothesis, and the results are shown in the table.

From the results of the correlation analysis of perceived susceptibility, perceived severity, perceived benefit, perceived barriers, and COVID-19 vaccination intention, the coefficients are 0.285^*∗∗*^, 0.305^*∗∗*^, 0.572^*∗∗*^, and −0.221^*∗∗*^, respectively, with the four groups of variables significantly correlated at the *p* < 0.01 level, while none of the correlation coefficients exceeded 0.8, so there was no colinearity between the four groups of variables and they were significantly correlated with COVID-19 vaccination acceptance, tentatively proving the validity of the four hypotheses (H5, H6, H7, H8). Regression analysis can be continued (Table 7).

### 3.5. Regression Analysis

Regression analysis of health beliefs and COVID-19 vaccination acceptance was performed. From *R*^2^ = 0.34, the independent variables are “perceived impairment,” “perceived benefit,” “perceived susceptibility,” and “perceived severity.” The equations explained 34% of the dependent variable “COVID-19 vaccination acceptance,” thus indicating a strong explanatory power within the acceptable range. The coefficient tables were further analyzed (Table 8).

“Perceived susceptibility,” “perceived severity,” and “perceived benefit” can well explain the propensity to receive the COVID-19 vaccine with high (*p* < 0.05); “perceived susceptibility” was positively correlated with “COVID-19 vaccination acceptance” (*β* = 0.12); “perceived severity “was positively correlated with “COVID-19 vaccination acceptance” (*β* = 0.10); “perceived benefit”was positively correlated with “COVID-19 vaccination acceptance” (*β* = 0.45); and “perceived impairment” was negatively correlated with “COVID-19 vaccination acceptance” (*β* = −0.133) (Table 9).

Thus, we addressed Q2 and concluded that different dimensions of health beliefs can have an impact on COVID-19 vaccine intention, and the hypotheses H5, H6, H7, and H8 are verified to hold.

## 4. Discussion

In this study, the reliability test, validity test, descriptive statistical analysis, Kruskal–Wallis H nonparametric test, correlation analysis, and regression analysis were conducted on 525 valid questionnaire data for two research questions and four research hypotheses. This study analyzed the effects of three major health information channels on the health beliefs of the COVID-19 vaccination-appropriate population and the effects of health beliefs on the intention to receive the COVID-19 vaccine and localized the health belief model in Beijing, China. To a certain extent, it expands the dimensions of health belief model studies and COVID-19 vaccine diffusion studies and enriches the study of health communication effects.

1. The audiences who mainly use new media communication channels as the main information receiving channels are the largest. Descriptive statistics showed that the three main health information receiving channels, namely, new media channels, interpersonal communication channels, and traditional media communication channels, all had a wide audience, with the broadest audience (45.5%) primarily using new media channels as the main COVID-19 vaccine information receiving channel and a relatively small audience (29.9%) using interpersonal communication channels as the main COVID-19 vaccine information receiving channel. Among several subchannels of interpersonal communication, communication with medical workers accounted for the highest percentage (65.29%) as the most critical channel of interpersonal communication of COVID-19 vaccine health information. Compared with traditional media communication channels and interpersonal communication channels, new media channels have many advantages. First, users can retrieve information more quickly and get information released by multiple subjects, which is good for analyzing information; second, on media platforms and news apps, more vaccine information is received passively in the form of the “trending hashtag.”
2. There are significant differences in perceived benefits and perceived barriers among the main audiences of the three information channels. There were differences in the health beliefs of audiences who chose interpersonal communication channels, new media channels, and traditional media communication channels, and the differences in perceived benefits and perceived barriers were significant. The perceived benefits of audiences in the interpersonal communication channel were higher and the perceived barriers were significantly lower than those of main audiences in the other two channels, and the perceived benefits and perceived barriers were key variables explaining the propensity to receive the COVID-19 vaccine. The test results found that the perceived barriers of the audience were higher in the new media channel, and the largest percentage of respondents used the new media channel as the main information acquisition channel, but its performance in influencing the perceived benefit and perceived hindrance of the audience needs to be optimized. Therefore, in the popularization of the COVID-19 vaccine, we should pay attention to the influence of inaccurate health information and redundant content on the perceived barriers of audiences in new media information dissemination and pay attention to the strength and breadth of scientific and systematic interpretation of content in new media channels. Moreover, the positive influence of interpersonal communication factors on the audience's health beliefs should be fully considered in the health communication of COVID-19 vaccine information. The positive influence of the subdivision channel of communication with medical personnel, an important component of interpersonal communication, should be paid attention to in the various forms of vaccine popularization by health organizations, community hospitals, and other staff medical workers.
3. Perceived benefits and perceived barriers have the highest explanatory power for COVID-19 vaccination acceptance. The results of the study suggest that perceived benefit and perceived barriers to vaccination are the two most important HBM dimensions influencing intention towards the COVID-19 vaccine. High perceived susceptibility to infection with COVID-19 and high perceived severity were also associated with increased intention to vaccinate in multivariate analyses. Thus, public health intervention programs should focus on increasing awareness of the benefits of vaccination and the perceived susceptibility and severity of infection while reducing concerns and possible obstacles to vaccination. The findings help influence vaccine-related behaviors. It is shown that audiences are more motivated to act when they recognize the benefits of COVID-19 vaccination and dispel doubts about negative barriers to vaccination. Therefore, when promoting COVID-19 vaccine-related health information, emphasis should be placed on information about the beneficial nature of COVID-19 vaccination and on reducing people's concerns about the negative impact of untrue vaccination. It is important to give full play to the role of traditional media, new media, and interpersonal communication channels in health communication.

## 5. Conclusion

Based on the exploration above, in the future, we should develop more appropriate vaccine promotion strategies under the background of a digital information society. First, governments and health departments should release comprehensive and authoritative information through multiple channels, so that the dissemination of vaccination awareness can be mutually reinforcing. Meanwhile, it could also maximize the efficiency of dissemination by regulating public sentiment and guiding rational vaccination behavior. It is also noted that inaccurate health information and redundant content in new media information dissemination channels, such as websites and social media, impact audience perception barriers. More efforts can be made to provide suggestions for reliable information sources for new media channels. In the health communication of COVID-19 pneumonia vaccine information, the positive influence of interpersonal communication factors on audience health beliefs should be fully considered, and attention should be paid to various forms of vaccine dissemination by healthcare workers, such as health organizations and community hospitals. School health education and various forms of vaccine dissemination by community-based health organizations, community hospitals, and other healthcare workers can be strengthened for interpersonal communication channels. For example, community healthcare workers in the United States and Hong Kong, China, have effectively increased prosocial vaccination by protecting vulnerable patients and the elderly [41]. Future attention should also be paid to applying new media technologies, such as virtual reality, in vaccination promotion, as the first-person experience of vaccination in immersive VR increases collective responsibility and vaccination intention more than pictures and text [42].

The HBM-based analysis showed that perceived benefits and barriers to vaccination had the highest predictive power for the public's propensity to receive vaccination against Neocon, so public health intervention programs should focus on increasing awareness of the benefits of vaccination. Also, reduce identified barriers and public concern about false side effects of vaccination. Government departments should target people with vaccination awareness bias, mobilize all parties to strengthen psychological counseling efforts comprehensively, and provide good humanistic care so that they can change their cognitive bias and resistance to the COVID-19 vaccination, stop continuing to spread rumors and tensions about the COVID-19 vaccination, and promote the formation of correct perceptions of COVID-19 vaccination among the community. At the same time, the price of vaccines may be an essential barrier to accepting self-pay vaccines [43, 44]. National governments should try to compensate for this by offering policies including free vaccination. For example, the governments of China, Japan, and other countries are providing the public with free COVID-19 vaccines and booster shots.

This study has highlighted the attributes of finding a relationship between information dissemination channels, health beliefs, and COVID-19 vaccination intention. Moreover, this work can provide a framework and theoretical basis for further research studies on this topic, especially in analyzing public perception and acceptance of the COVID-19 vaccine and COVID-19 booster vaccination and designing effective and appropriate vaccination expansion strategies when booster vaccines are widely recommended in the future.

## Figures and Tables

**Figure 1:** Relationship model diagram of information channels, health beliefs, and COVID-19 vaccination acceptance.

**Table 1:** Results of reliability analysis of “COVID-19 vaccination acceptance” and “health beliefs.”

Dimension	Cronbach's alpha	Cronbach's alpha terms based on normalized terms	Number of items
“COVID-19 vaccination acceptance”	0.954	0.956	3
Perceived susceptibility	0.620	0.669	4
Perceived severity	0.883	0.885	4
Perceived benefits	0.861	0.874	4
Perceived barriers	0.872	0.873	4

**Table 2:** Rotated component matrix of “health beliefs.”

	Ingredients			
	1	2	3	4
(7) I believe that contracting COVID-19 will threaten my lifelong happiness	0.872			
(6) I believe that infection with COVID-19 threatens my family relationships	0.845			
(8) I believe that infection with COVID-19 threatens my life	0.795			
(5) I think that infection with COVID-19 poses a serious threat to my daily activities (including work, contact with family and friends, and shopping)	0.717			
(14) I think that getting the COVID-19 vaccine will take a lot of my time and energy		0.871		
(15) I am afraid of the pain associated with vaccination		0.847		
(13) Getting information about COVID-19 vaccine will take a lot of my time and energy		0.840		
(16) I am afraid of the possible side effects of COVID-19 vaccination		0.818		
(9) Getting the COVID-19 vaccine will protect me from getting the new coronavirus			0.850	
(11) COVID-19 vaccination can improve the safety of daily social activities (including work, socializing with family and friends, and shopping)			0.811	
(10) The COVID-19 vaccination will protect me against the mutated COVID-19			0.770	
(12) In general, I think COVID-19 vaccination is beneficial			0.729	
(2) I think I may get a new coronavirus in the future if I am not protected				0.767
(3) I think that many people are at risk of contracting COVID-19, including my family, partner, and friends				0.744
(1) I think that anyone can get COVID-19 if they do not take the right personal precautions				0.698
(4) I think that I am more likely to get COVID-19 in the future				0.576
Cumulative variance explained (%)	33.90	52.92	61.68	69.26

Extraction method, principal component analysis; Rotation method, Kaiser normalized maximum variance method. Rotation has converged after 5 iterations.

**Table 3:** Exploratory factor analysis of “COVID-19 vaccination acceptance.”

	Ingredients
	1
(17) I will consider COVID-19 vaccination	0.975
(18) I plan to receive the COVID-19 vaccine	0.957
(19) I believe I will definitely receive the COVID-19 vaccine	0.944
Total variance explained rate	91.969

**Table 4:** Summary of basic information.

Demographic variables	Statistical variables	Frequency	Percentage
Gender	Male	231	44.0
	Female	294	56.0

Age (years)	16–25	176	33.5
	26–35	166	31.6
	35–45	145	27.6
	46–59	38	7.2

Education level	Under college	201	38.3
	Undergraduate	171	32.6
	Master's degree and above	153	29.1

Nature of work	Domestic school teachers, students	148	28.1
	Those who are going to work or study in medium- and high-risk countries or regions	5	0.9
	Staff working in import cold chain, port quarantine, ship pilotage, aviation aircrew, fresh market, public transportation, medical disease control, etc. with relatively high risk of infection	46	8.7
	General practitioners	178	33.9
	Farmers, migrant workers	80	15.2
	Retired employees	31	5.9
	Housewives	9	1.7
	Others	28	5.3

Main information	Interpersonal communication	127	24.2
	New media	239	45.5
	Traditional media	159	29.9

**Table 5:** Kruskal–Wallis H nonparametric test statistics for communication channels and health beliefs.

	Perceived susceptibility	Perceived severity	Perceived benefit	Perceived barriers
*K* ^2^	41.301	45.296	43.499	41.973
Degrees of freedom	2	2	2	2
Asymptotic significance (two-tailed)	0.127	0.061	0.000	0.000

Subgroup variables: 24. The main channels through which COVID-19 vaccine information were obtained are interpersonal communication, new media communication, and traditional media communication.

**Table 6:** Statistics of rank mean test for “perceived benefits” and “perceived barriers.”

(24) Your main source of information about COVID-19 vaccine		Number of cases	Rank average
Perceived benefits	Interpersonal communication channels	127	308.94
	New media channels	239	221.51
	Traditional media channels	157	277.83

Perceived barriers	Interpersonal communication channels	127	202.76
	New media channels	239	302.08
	Traditional media channels	157	259.80

**Table 7:** Pearson's correlation coefficient between “COVID-19 vaccination acceptance” and “health beliefs.”

		Perceived susceptibility	Perceived severity	Perceived benefit	Perceived barriers
COVID-19 vaccination acceptance	COVID-19 vaccination acceptance Pearson correlation	0.284^*∗∗*^	0.354^*∗∗*^	0.503^*∗∗*^	−0.221^*∗∗*^
	Significance (two-tailed)	0.000	0.000	0.000	0.000
	Number of cases	525	525	525	525

^*∗∗*^At the 0.01 level (two-tailed), the correlation is significant.

**Table 8:** Summary of the COVID-19 vaccination acceptance and the health beliefs model.

Model	*R*	*R* ^2^	Adjusted *R*^2^	Error in standard estimation	Durbin–Watson
1	0.583a	0.34	0.324	1.10501	1.961

Predictor variables: (constant), perceived barriers, perceived benefit, perceived susceptibility, perceived severity. Dependent variable: intention to vaccinate with COVID-19.

**Table 9:** Coefficients of the “COVID-19 vaccination acceptance” and “health beliefs” model.

Models		Unstandardized factor	Standardization factor		*t*	Saliency	Covariance statistics	
		*B*	Standard error	Beta			Tolerances	VIF
1	(Constant)	2.687	0.326		2.077	0.000		
	Perceived susceptibility	0.12	0.053	0.077	0.845	0.031	0.714	1.294
	Perceived severity	0.10	0.061	0.112	1.179	0.015	0.643	1.402
	Perceived benefit	0.45	0.053	0.385	7.142	0.000	0.655	1.307
	Perceived barriers	−0.133	0.032	−0.157	−1.064	0.000	0.945	1.101

Dependent variable, intention to receive COVID-19 vaccine.

## Data Availability

The Web of Science (WoS) data can be accessed through the WoS's official website: https://www.webofscience.com/wos/alldb/basic-search.
